# Effectiveness of Comprehensive Nursing in Hemodialysis of Patients with Chronic Renal Failure and the Impact on Their Quality of Life

This article has been retracted.

**DOI:** 10.1155/2022/1399650

**Published:** 2022-08-05

**Authors:** Quan Wen, Shuang Yao, Bingnan Yao

**Affiliations:** ^1^Songbei Nucleic Acid Clinic, Fourth Affiliated Hospital of Harbin Medical University, Harbin 150028, Heilongjiang, China; ^2^The Second Department of Hemodialysis, Fourth Affiliated Hospital of Harbin Medical University, Harbin 150028, Heilongjiang, China

## Abstract

**Objective:**

To assess the effectiveness of comprehensive nursing in patients with chronic renal failure undergoing hemodialysis and the impact on their quality of life.

**Methods:**

The present study included 86 patients undergoing hemodialysis for chronic renal failure from January 2020 to October 2021 and randomly assigned them to receive either normal nursing or comprehensive nursing, with 43 cases in each group. Outcome measures included psychological status, treatment compliance, quality of life, and complications of the eligible patients.

**Results:**

After the intervention, comprehensive nursing resulted in lower Self-Rating Anxiety Scale (SAS) scores and Self-Rating Depression Scale (SDS) scores and higher quality of life scores for patients versus routine nursing (*P* < 0.05). Comprehensive nursing was associated with a significantly higher overall patient compliance rate versus routine nursing (*P* < 0.05). Patients receiving comprehensive nursing had a lower risk of developing complications versus those given routine nursing (*P* < 0.05).

**Conclusion:**

Comprehensive care increases treatment compliance and self-care capacity of patients undergoing hemodialysis for chronic renal failure, improves their quality of life, and lowers the risk of complications, indicating a high potential for clinical advancement.

## 1. Introduction

Chronic renal failure [1] is secondary to the continuous progression of various chronic kidney diseases and is characterized by renal insufficiency, metabolite retention, dysregulation of the internal environment, and functional imbalance of systems. Clinical statistics show that the annual incidence of chronic renal failure is about 0.3%, which exhibits an increasing trend in recent years, and the incidence of chronic kidney disease in Chinese adults is about 10.8% [2, 3]. Patients with chronic renal failure have exceedingly complicated clinical symptoms that may be split into two categories: metabolic abnormalities and systemic multisystem symptoms. The majority of individuals with stages I–III are asymptomatic or present moderate symptoms such as fatigue, anorexia, and mild anemia. Disease progression is associated with more severe symptoms such as heart failure, hyperkalemia, gastrointestinal bleeding, and neurological disorders, posing a great threat to the health of patients [4]. Evidence has confirmed the association of the occurrence of chronic renal failure with primary glomerular disease, diabetic nephropathy, immune disease kidney damage, and drug-related kidney damage; besides, the disease progression is accelerated in the presence of infection, insufficient blood circulation, and the use of nephrotoxic drugs [5]. Hemodialysis [6] is a renal replacement therapy for acute and chronic renal failure, which effectively removes metabolites and toxic substances from the body, maintains the balance of water electrolytes and acidity [7, 8], discharges excess water from the body, and substantially improves prognosis [9]. According to the findings of relevant research, hemodialysis alleviated patients' symptoms and improved their quality of life within 6 weeks of therapy. Nonetheless, the condition is prone to recurrence, whereas long-term hemodialysis is associated with physical discomfort. Patients with chronic renal failure are predisposed to negative emotions such as anxiety and depression, which compromise treatment compliance and treatment effect. Clinical treatment of the disease highlights the treatment of the primary cause, avoidance of risk factors, prevention of complications, and substitution therapy, and the formulation of treatment protocols entails the integration of factors such as primary illness and symptoms. Moreover, the recurrence of the disease causes inconvenience to patients and their families and further triggers negative emotions such as anxiety [10, 11]. According to traditional Chinese medicine (TCM), chronic renal failure belongs to the categories of “edema,” “exertional labor,” and “retention of urine.” The long duration and the slow recovery of chronic renal failure impose a large financial burden on patients and severely compromise their quality of life [12]. Clinical findings indicate that effective care methods could reduce medical costs and improve patient satisfaction [13]. In China, the TCM care guideline for chronic renal failure was developed by the State Administration of Traditional Chinese Medicine in 2015 [14, 15]. Furthermore, research suggests that competent nursing care during hemodialysis aids disease recovery and improves patient prognosis [14, 15]. Comprehensive nursing systematizes nursing procedures, coordinates standardized nursing plans and nurse training programs, and integrates the advantages of accountable care and group nursing to ensure the quality of care [16]. As a result, from January 2020 to October 2021, patients undergoing hemodialysis for chronic renal failure in our hospital were recruited to analyze the effectiveness of comprehensive nursing in hemodialysis of patients with chronic renal failure and the influence on their quality of life.

## 2. Materials and Methods

### 2.1. Participants

A total of 86 patients undergoing hemodialysis for chronic renal failure in our hospital from January 2020 to October 2021 were recruited and assigned to receive routine nursing (control group) or comprehensive nursing (observation group) via the random number table method, with 43 cases in each group. Informed consent was obtained from patients and signed prior to enrollment in this study. The study protocol was approved by the hospital ethics committee, with an ethical number of JX-JUE20200104. All procedures complied with the Declaration of Helsinki's ethical guidelines for clinical research.

### 2.2. Inclusion and Exclusion Criteria

Inclusion criteria: patients with diagnosis of chronic renal failure confirmed by relevant examinations, who received hemodialysis for ≥3 months, and who provided written informed consent were included.

Exclusion criteria: patients with infections, cardiovascular diseases, and other related diseases, with other serious medical diseases, with coagulation disorders, or with an abnormal mental status that prevented normal communications were excluded.

### 2.3. Treatment Methods

All patients were treated with hemodialysis. Hemodialysis was performed under systemic heparinization using a polysulfone membrane high-flux dialyzer from B. Braun Avitum AG [17] with a dialysate flow of 500 ml/min and a blood flow of 200–300 ml/min. The duration of hemodialysis was 4 h each and was performed thrice a week.

The control group received routine nursing, including pre-dialysis preparation, weight measurement, basic health education, close monitoring of vital signs and conditions, dialysis machine management, and prevention of dialysis complications [18].

The observation group received comprehensive nursing. (1) Health education: The patients were educated about the knowledge of chronic renal failure and hemodialysis, treatment methods, and possible complications. (2) Dietary guidance: The nutritional indices, renal function, water, and electrolytes were analyzed, and the nutritional status of the patients was evaluated according to their condition. Patients were instructed to follow a diet high in protein, low in salt, and low in phosphorus foods during treatment and were prohibited from any potassium-containing foods. Patients and their families were informed of the causes and consequences of malnutrition, with emphasis on the importance of reasonable intake of energy, water, protein, sodium, potassium, and phosphorus. (3) Dialysis care: Prior to dialysis, the nursing staff informed the patients of the dialysis process and precautions, as well as the potential issues of dialysis. Patients' vital signs were continuously monitored throughout dialysis, and the functioning of the dialysis equipment, as well as the condition of the dialysis catheter, dialysis fluid, and blood, was meticulously documented. The doctor was timely informed in terms of abnormalities of the patients. After dialysis, the puncture site was disinfected with 75% alcohol and warmed with hot towels to prevent adverse reactions such as swelling and pain. (4) Psychological intervention: The nursing staff relieved patients' negative emotions through positive psychological guidance, emotional reassurance, and other nursing measures to enhance their treatment compliance and confidence. (5) Daily care: Daily plans were developed based on the patients' actual postoperative conditions, such as out-of-bed activities and nutrition instructions. Both groups were intervened for 3 months.

### 2.4. Outcome Measures

1. Negative emotions: Self-Rating Anxiety Scale (SAS) and Self-Rating Depression Scale (SDS) [19, 20] were used to assess the emotional status of patients. Both scales have 20 items each with a total score of 100, with 50–70 for mild anxiety/depression, 71–90 for moderate anxiety/depression, and >90 for severe anxiety/depression. The higher the score, the higher the degree of anxiety/depression of the patient.
2. Compliance: The “Exercise Adherence Scale” created by our hospital was used for the compliance evaluation, which was divided into full compliance, partial compliance, and noncompliance. The total score of the scale was 10 points, with ≥8 for complete compliance, 6–8 for partial compliance, and <6 for noncompliance. The total compliance rate was calculated and compared between the two groups. Total compliance rate = (complete compliance + partial compliance)/total number of cases × 100%.
3. Quality of life: The MOS 36-item short-form health survey (SF-36) [21] was used to assess the quality of life of patients, which included five domains of physical function, emotional function, role function, social function, and cognitive function, with a total score of 100 points for each domain. Higher scores indicated higher quality of life for patients.
4. Complications: The occurrence of complications, such as bleeding, infection, hypotension, nausea and vomiting, and cardiac arrhythmias, was meticulously documented for all patients, and the total incidence of complications was computed and compared individually for the two groups.

### 2.5. Statistical Analysis

SPSS22.0 was used for data analyses. The measurement data were expressed as ($\bar{x}\pm s$) and analyzed using the independent sample *t*-test. The count data were expressed as cases (%) and analyzed using the chi-square test. *P* < 0.05 was used as a cutoff for statistical significance.

## 3. Result

### 3.1. Patient Characteristics

In the observation group, there were 43 patients, 25 males and 18 females, aged 38–69 (50.04 ± 5.17) years, with 12 cases of diabetic nephropathy, 17 cases of chronic glomerulonephritis, and 14 cases of hypertensive nephropathy. In the control group, there were 43 patients, 24 males, and 19 females, aged 35–70 (49.79 ± 5.08) years, with 13 cases of diabetic nephropathy, 17 cases of chronic glomerulonephritis, and 13 cases of hypertensive nephropathy. The duration of disease in the control group was (2.42 ± 0.79) years and in the observation group was (2.14 ± 1.17) years. The patient characteristics of the two groups were comparable (*P* > 0.05) (Table 1).

### 3.2. Negative Emotions

Prior to the nursing care, the difference in negative emotions between the two groups was not statistically significant (*P* > 0.05). After the intervention, comprehensive nursing resulted in lower SAS scores and SDS scores (40.17 ± 3.18, 45.85 ± 3.26) versus routine nursing (51.01 ± 3.45, 57.08 ± 4.32) (*P* < 0.05) (Table 2).

### 3.3. Treatment Compliance

The number of completely and partially complying patients in the observation group (19, 23) was substantially greater than in the control group (13, 19), whereas the number of noncompliant patients (1) was significantly lower than that in the control group (11). Comprehensive nursing was associated with a significantly higher overall patient compliance rate versus routine nursing (*P* < 0.05) (Table 3).

### 3.4. Quality of Life

Prior to the intervention, there was no statistically significant difference in the two groups' quality of life scores (*P* > 0.05). Comprehensive nursing resulted in considerably superior quality of life ratings, including physical function, emotional function, role function, social function, and cognitive function scores after nursing (69.47 ± 6.11, 74.36 ± 5.94, 68.96 ± 6.03, 65.24 ± 6.14, 72.87 ± 5.91) versus routine nursing (57.57 ± 6.17, 64.56 ± 4.99, 55.56 ± 6.23, 57.98 ± 5.96, 60.58 ± 5.48) (*P* < 0.05) (Table 4).

### 3.5. Complications

In the observation group, there were 0 (0.00%) cases of bleeding, 1 (2.33%) case of infection, 1 (2.33%) case of hypotension, 2 (4.65%) cases of nausea and vomiting, and 0 (0.00%) cases of cardiac arrhythmia. In the control group, there were 2 (4.65%) cases of bleeding, 4 (9.30%) cases of infection, 3 (6.98%) cases of hypotension, 5 (11.63%) cases of nausea and vomiting, and 2 (4.65%) cases of arrhythmia. Comprehensive nursing was associated with a lower complication rate (9.30%) versus routine nursing (37.21%) (*P* < 0.05) (Table 5).

## 4. Discussion

Chronic renal failure is a clinical syndrome caused by various chronic kidney diseases [22] and is characterized by an imbalance of water, electrolytes, and acidolysis. Disease progression may lead to complete loss of renal function and uremia [23]. Hemodialysis is the preferred treatment for chronic renal failure and is effective in improving patient prognoses [24]. However, the prolonged duration of hemodialysis is associated with increased stress and complications in patients during treatment, resulting in a compromised prognosis [25]. To the best of our knowledge, specific drugs for chronic renal failure are still not available in modern medicine even in the early and middle stages of the disease. Therefore, great attempts have been devoted in recent years to seek breakthroughs in TCM treatment methods. Modern pharmacological studies of TCM have demonstrated that Radix Codonopsis and Radix Astragali could regulate immunity, reduce urinary protein, and protect the kidney [26, 27]; salvia and Angelica could inhibit fibroblast proliferation and modify renal capillary permeability in the treatment of membranous nephropathy [28, 29]; the active ingredients of earthworm [30] could prevent platelet aggregation, inhibit vasoconverting enzyme activity and renal interstitial fibrosis, and protect renal function. Relevant clinical research has shown that effective nursing care during hemodialysis for patients with chronic renal failure could reduce complications and improve patients' quality of life and prognosis [31].

The TCM care protocol for chronic renal failure emphasizes the holistic view of TCM and the guiding ideology of evidence-based care, whereby “different care for the same disease” and “same care for different diseases” are incorporated to provide patients with evidence-based care in terms of daily living, diet, mood, and medication care [32]. For example, moxibustion stimulates acupuncture points or painful areas through the warmth and medicinal effects of moxa to warm the meridians, disperse cold, support Yang, consolidate detachment, and tonify kidney energy. Ear acupressure with Vaccariae Semen applied to acupuncture points on the auricle ameliorates lumbar and knee weakness through meridian stimulation and adjusts the qi and blood functions of the internal organs [33]. As a result, from January 2020 to October 2021, patients with chronic renal failure undergoing hemodialysis in our hospital were recruited to analyze the effectiveness of comprehensive nursing in hemodialysis of patients with chronic renal failure and the influence on their quality of life.

The results of the present study showed that comprehensive care resulted in significantly lower SAS and SDS scores versus routine care. Negative emotions during the long duration of hemodialysis in patients may undermine patient compliance and reduce dialysis outcomes, while previous conventional hemodialysis care is less targeted to the nursing of patients' negative emotions [34]. Comprehensive care strengthens patients' understanding of kidney disease and dialysis treatment, and targeted psychological interventions mitigate the negative emotions of patients, thereby increasing treatment compliance. The results showed that patients in the observation group had a higher overall compliance rate (97.67%) than that of the control group (74.42%), and the quality of life scores of the observation group were higher than those of the control group. Comprehensive care is designed to improve patients' disease awareness and increase their treatment proactiveness to enhance the therapeutic and nursing effects. With the aforementioned results of this study, the application of comprehensive nursing care to patients with chronic renal failure during hemodialysis could effectively mitigate the negative emotions of patients, thereby increasing their treatment compliance and improving their quality of life. Nevertheless, relevant clinical data show that maintenance hemodialysis prolongs the survival time of patients with renal failure by more than 15–20 years, but its extended treatment duration and susceptibility to recurrent episodes are associated with physical discomfort and complications, posing a serious threat to patient prognosis and quality of life. The results herein showed that patients in the observation group had a lower overall incidence of complications (9.30%) than the control group (37.21%), suggesting that the application of comprehensive care for patients with chronic renal failure during hemodialysis could effectively lower the risk of complications in patients. The reason for this is because comprehensive care offers patients integrated treatment including basic evaluation, psychological care, health education, skincare, and nutritional care. Comprehensive nursing for hemodialysis patients has been indicated to be advantageous in increasing patient compliance and clinical outcomes, improving quality of life, and extending patient longevity, which is consistent with the current study's findings.

According to the current treatment status, the combination of TCM care may be contributory to better efficacy, such as TCM enema, acupressure, TCM ionization, and topical application. Future studies with a larger sample size and integration of TCM nursing will be conducted to reinforce the current conclusion.

## 5. Conclusion

Comprehensive care increases treatment compliance and self-care capacity of patients undergoing hemodialysis for chronic renal failure, improves their quality of life, and lowers the risk of complications, indicating a high potential for clinical advancement.

## Figures and Tables

**Table 1:** Patient characteristics ($\bar{x}\pm s$, %).

Group	*n*	Gender		Age		Underlying disease		
		Male	Female	Range	Mean	Diabetic nephropathy	Chronic glomerulonephritis	Hypertensive nephropathy
Observation	43	25	18	38–69	50.04 ± 5.17	12 (27.91)	17 (39.53)	14 (32.56)
Control	43	24	19	35–70	49.79 ± 5.08	13 (30.23)	17 (39.53)	13 (30.23)
*t*-value	—	0.047		—	0.226	0.056	0.000	0.054
*P*-value	—	0.828		—	0.822	0.812	1.000	0.816

**Table 2:** SAS and SDS scores ($\bar{x}\pm s$).

Group	*n*	Before intervention (point)		After intervention (point)	
		SAS	SDS	SAS	SDS
Observation	43	68.94 ± 2.96	69.98 ± 2.36	40.17 ± 3.18^*∗*^	45.85 ± 3.26^*∗*^
Control	43	69.05 ± 2.82	69.74 ± 2.44	51.01 ± 3.45^*∗*^	57.08 ± 4.32^*∗*^
*t*-value	—	0.176	0.4 64	15.150	13.607
*P*-value	—	0.861	0.644	<0.001	<0.001

*Note.* ^*∗*^ indicates a significant difference between pre- and posttreatment data in the same group.

**Table 3:** Treatment compliance (%).

Group	*n*	Full compliance	Partial compliance	Noncompliance	Compliance rate
Observation	43	19 (44.19)	23 (53.49)	1 (2.33)	42 (97.67)
Control	43	13 (30.23)	19 (44.19)	11 (25.58)	32 (74.42)
*x* ^2^	—	9.685			
*P*	—	0.002			

**Table 4:** Quality of life ($\bar{x}\pm s$).

Time	Domains	Observation (*n* = 43)	Control (*n* = 43)	*t*-value	*P*-value
Before nursing	Physical function	45.56 ± 5.23	45.87 ± 5.65	0.264	0.792
	Emotional function	53.41 ± 5.45	53.26 ± 5.24	0.101	0.897
	Role function	48.51 ± 5.54	48.17 ± 5.74	0.274	0.781
	Social function	50.15 ± 5.96	50.44 ± 5.11	0.242	0.809
	Cognitive function	54.92 ± 5.27	55.03 ± 5.08	0.099	0.921

After nursing	Physical function	69.47 ± 6.11^*∗*^	57.57 ± 6.17^*∗*^	8.987	<0.001
	Emotional function	74.36 ± 5.94^*∗*^	64.56 ± 4.99^*∗*^	8.284	<0.001
	Role function	68.96 ± 6.03^*∗*^	55.56 ± 6.23^*∗*^	10.135	<0.001
	Social function	65.24 ± 6.14^*∗*^	57.98 ± 5.96^*∗*^	5.564	<0.001
	Cognitive function	72.87 ± 5.91^*∗*^	60.58 ± 5.48^*∗*^	9.999	<0.001

*Note.* ^*∗*^ indicates a significant difference between pre- and posttreatment data in the same group.

**Table 5:** Complications (%).

Groups	*n*	Bleeding	Infection	Hypotension	Nausea and vomiting	Cardiac arrhythmia	Total incidence
Observation	43	0 (0.00)	1 (2.33)	1 (2.33)	2 (4.65)	0 (0.00)	4 (9.30)
Control	43	2 (4.65)	4 (9.30)	3 (6.98)	5 (11.63)	2 (4.65)	16 (37.21)
*x* ^2^	—	9.382					
*P*-value	—	0.002					

## Data Availability

All data generated or analyzed during this study are included in this published article.
